The article "Concurrent Hearing and Genetic Screening among Newborns in Ningbo, China" was retracted in 2023. Reasons: signs of a paper mill; compromised peer review; unreliable results or conclusions.

# Concurrent Hearing and Genetic Screening among Newborns in Ningbo, China

**DOI:** 10.1155/2022/1713337

**Published:** 2022-01-10

**Authors:** Cao Guomei, Zhang Luyan, Dai Lingling, Huang Chunhong, Chen Shan

**Affiliations:** ^1^Department of Laboratory Medicine, Ningbo Mingzhou Hospital, Ningbo 315000, China; ^2^Beijing CapitalBio Technology, Beijing 101111, China; ^3^Department of Obstetrics, Ningbo Mingzhou Hospital, Ningbo 315000, China

## Abstract

**Objective:**

To detect the carrier rates of deafness gene variants in populations in Ningbo and analyze the risk of hereditary hearing loss through concurrent hearing and genetic screening tests.

**Methods:**

Two thousand one hundred and seventy-four newborns were enrolled from November 2018 to August 2019. All subjects underwent hearing screening and newborn deafness genetic screening with 15 variants in 4 genes, and the positive sites were simultaneously verified by sequencing.

**Results:**

The total carrier rate of genetic variants in Ningbo reached 4.32%, when *GJB2* c.235delC was the variant with the highest prevalence (2.12%), approximately accounting for 48.9% of the total carrier frequency. The carrier frequency of *SLC26A4* c.919-2A>G was 0.87%, while the most common variant in mitochondrial DNA (mtDNA) *MT-RNR1* gene was m.1555A>G, and its carrier frequency was 0.184%. In the OAE testing, 92 newborns passing hearing screening were tested positively for variants in 4 genes, and 2 of 42 newborns who failed in the first hearing test were found to mutate in 4 genes.

**Conclusion:**

Herein, the results concerning the carrier rates for deafness gene mutations of Ningbo population are reported. Our study is beneficial to the insight into the deafness genomic epidemiology for deafness genes in Ningbo population and provides the reference for healthcare in Ningbo.

## 1. Introduction

Hearing loss has become a popular illness worldwide that severely endangers people's life quality. In the last few decades, 27.8 million cases of hearing loss, making up a proportion of 33.5% of the total disability, have been reported in China [1–3]. Furthermore, there will be 35,000 new congenital deaf children every year, and the deaf children caused by unreasonable use of antibiotics and environmental factors in China are also increasing at the rate of 30,000-50,000 per year, especially in underdeveloped regions [2–4].

Heredity is the biggest cause of hearing loss, and more than 60% of hearing loss patients are related to hereditary deafness genes [4]. Since 2003, the molecular diagnosis center of deafness in PLA general hospital has taken the lead in conducting a nationwide investigation on the molecular epidemiology of hearing loss. The results show that *GJB2*, *SLC26A4*, mitochondrial genes, and *GJB3* as well as other genes constitute the most prevalent deafness genes of China [4].

The article "Concurrent Hearing and Genetic Screening among Newborns in Ningbo, China" was retracted in 2023. Reasons: signs of a paper mill; compromised peer review; unreliable results or conclusions.

Universal newborn hearing screening is one of the important strategies for early detection and diagnosis of hearing impairment, but it has its own limitations. As for delayed hearing loss, drug-induced hearing loss and other newborns who do not show hearing loss at birth, they cannot be timely detected and predicted. Therefore, the combined screening of hearing and genetic deafness genes in neonates is a scientific means for early detection and intervention of delayed hearing loss and drug-induced hearing loss.

In our study, the leading mutation type and rate of four common deafness genes among the newborn in Ningbo were reported, and at the same time, the significance of concurrent hearing testing and genetic screening in a large-scale manner was presented.

## 2. Method

### 2.1. Subjects

Totally, 2174 newborns were enrolled from November 2018 to August 2019 in Mingzhou Hospital of Zhejiang University. And the selected cases were all Han Chinese neonates from Ningbo who were to be born in our hospital. The otoacoustic emission (OAE) test and genetic screening were concurrently performed in infants. Besides, all parents had been inquired for a full history and presented a written informed consent prior to the research, while doctors and genetic counselors took charge of explaining screening outcomes and then raising feasible intervening measures for mutation carriers. Here, it should be noted that the research had obtained approval from the institutional review board at Mingzhou Hospital of Zhejiang University.

### 2.2. Sample Collections and Genomic DNA Extraction

Three blood spots with the diameter of no less than 8 mm were gathered from the heel venous blood in the newborn within 3 days after birth. Then, they were naturally dried and stocked in preparation. Apart from that, the whole blood genomic DNA extraction system kit (No. 360100-01, Chengdu Biotech, China) was adopted, while DNA concentration was 3–25 ng/*μ*l, and DNA purity (OD 260/280) reached 1.7–2.0.

### 2.3. Array for the Mutation Screening

CapitalBio Gene Chip array kit (No. 300068) in deafness gene mutation detection, with approval from the National Medical Products Administration, was used in the study. Besides, simultaneous screening on the 4 genes (*GJB2*, *GJB3*, *SLC26A4*, and *MT-RNR1*) was made by adopting DNA microarray technology, when their mutations are c.35delG, c.176_191del16, c.235delC, c.299_300delAT; c.IVS7-2A>G, c.2168A>G, c.1174A>T, c.1226G>A,c.IVS15+5G>A, c.1975G>C, c.2027T>A, c.1229C>T; c.538C>T; and m.1555A>G, m.1494C>T. According to the protocol, 15 amplicons in the four genes were augmented using multiplex PCR technology. Then, the PCR reaction mixture had hybridization with specific tag probes fixed onto the microarray chip. Finally, chip signals were scanned and imaged using LuxScan Microarray Scanner and the detection system.

The article "Concurrent Hearing and Genetic Screening among Newborns in Ningbo, China" was retracted in 2023. Reasons: signs of a paper mill; compromised peer review; unreliable results or conclusions.

### 2.4. Sequencing

The genomic region for 4 genes having mutations was amplified with PCR, followed by sequencing using the ABI PRISM BigDye3.1 terminator cycle sequencing kit (ABI USA).

### 2.5. Hearing Screening

The OAE screening was performed using Madsen AccuScreen within 48-72 hours after neonatal birth. Then, newborns having abnormal OAE were tested repeatedly 42 days later, and hearing loss was verified through conducting brain auditory-evoked potential (BAEP) and further audiological diagnosis examinations by audiologists of the superior hospital, if the newborn still does not pass the second screening.

### 2.6. Statistical Analysis

The statistical analysis was made by IBM SPSS Statistics 20 statistical software. The *χ*^2^ or Fisher's exact test was performed in rate analysis, and *p* < 0.05 was statistically significant.

## 3. Results

### 3.1. Results of the Genetic Screening

Genetic screening data for 15 deafness-related loci from 4 genes can be seen from Table 1 and Figures 1 and 2. In the 2,174 newborns included by the research, 94 were tested positively for mutations from 4 common deafness genes. The total rate of genetic variants reached 4.32%. To be specific, 55 mutations were detected from *GJB2* gene, accounting for 2.53% in the tested newborns, while there were 3, 31, and 4 mutations detected from *GJB3*, *SLC26A4*, and *MT-RNR1* genes, respectively, with corresponding mutation rates of 0.18%, 1.43%, and 0.18%, accordingly (Table 1).

Among 2,174 newborns being tested, according to Table 1, 1 c.35delG case, 2 c.176_191del16 cases, 46 c.235delC cases, and 6 c.299_300delAT cases had heterozygous mutations, and carrier rates of *GJB2* mutations reached 0.05%, 0.09%, 2.12%, and 0.28% separately. Besides, 4 cases for c.538C>T heterozygous mutations from *GJB3* gene were detected, with corresponding detective rate of 0.18%. The c.2168A>G and c.IVS7-2A>G mutations from *SLC26A4* gene were found in 5 and 19 cases, respectively, with corresponding mutation rates of 0.28% and 1.08%. Additionally, 4 homozygous mutations were detected, with corresponding detective rate of 0.18%.

The total mutation frequency of the research was 4.32%. *GJB2* c.235delC was the variant with the highest prevalence (2.12%), accounting for approximately 48.9% of the total carrier frequency, while the carrier frequency of *SLC26A4* c.919-2A>G was 0.87%. In addition, the most frequent variant in *MT-RNR1* gene was m.1555A>G, and its carrier frequency was 0.184%.

The article "Concurrent Hearing and Genetic Screening among Newborns in Ningbo, China" was retracted in 2023. Reasons: signs of a paper mill; compromised peer review; unreliable results or conclusions.

### 3.2. Sequencing Validation

Mutations detected from 94 newborn samples were also verified by direct sequencing (Table 2 and Figure 3). The result suggested that the genetic chip method was feasible for screening deafness gene mutation.

### 3.3. The Hearing Screening Test and Mutations in the Four Common Deafness Genes in 2,174 Newborns

The OAE screening test was conducted on every newborn, when 42 cases failed to pass the first screening. Then, according to the secondary screening after 42 days of birth, 19 cases failed (Table 3). In addition, 1.93% (42/2174) newborns failing the initial hearing screening test received the second hearing screening test. Around 45% (19/42) of the newborns did not pass the hearing screening secondly. Apart from that, 2 of the 19 newborns failing the second hearing test accepted mutation testing, and the detective rate was 1.05% (see Tables 3 and 4). However, 94 of the 2174 newborns who underwent the hearing tests were tested positive for mutations in 4 genes. 2 of 19 newborns failing the hearing test were detected for mutations in 4 genes, composed of one case for *GJB2* c.299_300delAT heterozygous variant and one case for *SLC26A4* c.2168A>G heterozygous mutation (see Table 4).

## 4. Discussion

In this study, we report the results concerning the distribution of deafness gene mutations in Ningbo population. Besides, a comprehensive survey on newborns in a large scale is also conducted so as to detect the risk of hereditary hearing loss through concurrent hearing and genetic screening.

Genetic mutations from *GJB2*, *GJB3*, *SLC26A4*, and *MT-RNR1* genes have been considered as the most prevalent variants for hearing loss. The study shows that the mutation incidence rate in newborn screening for deafness gene mutations in Beijing, Wuhan, Southern China, and Northwest China is 4.508%, 4.51%, 2.976%, and 4.04% respectively [4–7]. Besides, the current research indicated the total mutation rate of Ningbo, Southeast China, is 4.32%, basically in agreement with that of other places in China. Moreover, the study here is the first newborn screening for gene mutations by 15 loci gene chips in Ningbo. It is also found that genes *GJB2* and *SLC26A4* have the highest mutation rates in comparison with the other places in China. Apart from that, our findings revealed the sites with the highest mutation rates, namely, c.235delC, c.IVS7-2A>G, c.299delAT, c.2168A>G, c.1174A>T, m.1555A>G, and c.538C>T, generally identical with other results of China.

*GJB2* gene is involved in the pathogenesis of autosomal recessive inherited nonsyndromic hearing loss, and the variant c.235delC is known to increase susceptibility to hereditary hearing loss [8]. *SLC26A4* and *GJB3* gene mutations do not necessarily cause phenotypic changes in early life, whereas newborns are likely to have progressive hearing loss [9]. Thus, people tested positive for genetic screening but negative for the hearing test should be focused on. Actually, c.IVS7-2 A>G mutation in *SLC26A4* gene is the main mutation site of the large vestibular aqueduct syndrome in the Chinese population. This study discovers that the detection rate of c.IVS7-2 A>G mutation in *SLC26A4* gene is the highest (1.53%), followed by c. 2168A> G, which is the same as the results in domestic literature [10]. Furthermore, studies have revealed that there are significant regional and ethnic differences in the site mutation of *SLC26A4* gene. For the Iranian population, *SLC26A4* c.1334T > G is the most common mutation, accounting for 10% of the study population [11]. In addition, due to the different screening methods of neonatal deafness genes in different regions of China, the mutation rate of deafness genes is not the same.

The article "Concurrent Hearing and Genetic Screening among Newborns in Ningbo, China" was retracted in 2023. Reasons: signs of a paper mill; compromised peer review; unreliable results or conclusions.

In this study, 4 cases of m.1555A>G homoplasmic mutation were detected. All of these cases passed the newborn hearing screening, but genetic screening results clearly indicated their sensitivity to aminoglycoside antibiotics. Thus, newborns with this gene mutation should avoid ototoxic antibiotics for their entire life. Moreover, the early research reported that the m.1555A>G homoplasmic mutation is among the major reasons of aminoglycoside-caused and nonsyndromic hearing loss [12].

The results suggested 92 of the 94 patients passed hearing screening tests, but they were tested positive for mutation screening. Patients experiencing mutations did not undergo hearing loss when they were young, but abnormal hearing might occur in their late life [13]. In addition, the 92 subjects with variants that passed the newborn hearing screening stated that 4.23% (92/2174) newborns would be benefited from genetic screening and possibly received better clinical intervention and management. Furthermore, our study underlined the clinical significance of both genetic and hearing screening. However, only 2 out of the newborns who failed the hearing screening were featured with variants, which may be due to the following two limitations. For one thing, there are only 15 mutations that were screened. Although they are the most common mutations, large-scale population screening has not been carried out in Ningbo, thus being unable to determine whether it is applicable. In addition, different hearing screening methods also have some limitations. For another, our sample size is limited, especially the abnormal sample being screened. The heterozygous mutations found in this study may not immediately cause hearing changes in infants [13], but the infants with hearing abnormalities need further genetic examination so as to identify the cause. Therefore, additional molecular genetic studies should be planned for the patients. In this case, in our study, it is suggested that whole exome/genome sequencing (WES/WGS) should be further performed.

The article "Concurrent Hearing and Genetic Screening among Newborns in Ningbo, China" was retracted in 2023. Reasons: signs of a paper mill; compromised peer review; unreliable results or conclusions.

The joint genetic screening of neonatal hearing and hereditary deafness provides a scientific means for early detection and intervention of delayed and drug-induced deafness. Universal newborn hearing screening is one of the effective strategies for early detection and diagnosis of hearing impairment. However, newborns who do not show hearing loss at birth, such as delayed and drug-induced deafness, cannot be detected and predicted in time, resulting in the omission. Neonatal deafness gene screening can not only detect children with congenital deafness caused by *GJB2* gene but also warn of large vestibular aqueduct syndrome caused by *SLC26A4* gene and drug-induced deafness caused by *MT-RNR1* gene, aiming to effectively prevent the occurrence of delayed deafness and drug-induced deafness.

In the research, the gene chip array was applied for approximately 5 h in every test. Thus, with cost-effective and rapid turnaround, the screening of large populations is feasible. Here, it should be noticed that the next-generation sequencing provides a stronger solution [10, 14],whereas organizing massive population genetic screening is challenging, which also increases interpretation burden. In addition, the microarray platform shows excellent detection sensitivity to the heteroplasmic mitochondrial variants. It can differentiate heteroplasmic variants of <5% of mtDNA *MT-RNR1*, while the next-generation sequencing cannot reach [4]. Other than that, subjects' samples are easy to be collected by blood spots and can be permanently preserved after drying. Therefore, the gene chip array belongs to a fast and easy-to-use genetic screening method applicable to population genetic diagnostics and follow-up [7, 15].

In conclusion, our research helps understand the deafness genomic epidemiology in Ningbo population and provides insight and evidence on healthcare in Ningbo. However, there are also some limitations. First, there is no enough large sample number of newborns with concurrent genetic and hearing screening. Second, although the hearing screening is passed, long-term follow-up is still required. Third, human cytomegalovirus (HCMV) infection is not planned in our research. HCMV screening might improve the detection for newborns with hearing loss risk but passing newborn hearing screening [16].

The article "Concurrent Hearing and Genetic Screening among Newborns in Ningbo, China" was retracted in 2023. Reasons: signs of a paper mill; compromised peer review; unreliable results or conclusions.

## Figures and Tables

**Figure 1:** The workflow of neonates' deafness gene screening.

**Figure 2:** Screening of genetic mutations in common deafness genes in newborns.

**Figure 3:** Validation of gene mutations by direct sequencing.

**Table 1:** Deafness gene mutation carrier rates detected in 2174 newborns.

Gene name	Site and nucleotide change	No. of cases	Heterozygous or homozygous	Carrier frequency (%)	Total rate (%)
*GJB2*	c.35delG c.176_191del16 c.235delC c.299_300delAT	1 2 46 6	Heterozygous Heterozygous Heterozygous Heterozygous	0.05 0.09 2.12 0.28	2.53
*GJB3*	c.538C>T	4	Heterozygous	0.18	0.18
*SLC26A4*	c.IVS7-2A>G c.2168A>G c.1174A>T c.1226G>A c.IVS15+5G>A c.2027T>A c.1229 C>T	19 5 5 1 0 0 0	Heterozygous Heterozygous Heterozygous Heterozygous	0.87 0.23 0.23 0.05	1.43
	c.1975G>C	1	Heterozygous	0.05	
*MT-RNR1*	m.1555A>G m.1494C>T	4 0	Homoplasmy	0.18	0.18

Comparison of the mutation rate in *GJB2* and *SLC26A4*, *χ*^2^ = 1.020, *p* = 0.312 (>0.05).

**Table 2:** Sequencing primers for four gene mutations.

Gene	Mutations	Primer names	Primer sequence (5′-3′)	Purification
*GJB2*	c.35delG, c.176_191del16, c.235delC, c.299_300delAT	F	CCCAGAGTAGAAGATGGATTG	PAGE
		R	CTTGATGAACTTCCTCTTCTTCT	
*GJB3*	c.538C>T	F	CTGCAGCTCATCTTCGTCACAT	PAGE
		R	TCGAGGCTTGTCCTTGTGCA	
*SLC26A4*	c.IVS7-2A>G	F	GTATGTAATGGTCTCTGTATCAA	PAGE
		R	GGAGTATCAGTGAAATGAAGCTT	
	c.2168A>G	F	CCTAGGAACTAACAAAACATTGTGTC	PAGE
		R	CTGTAGAAAGGTTGAATATTTACC	
	c.1174A>T, c.1226G>A	F	ATTTGTAGGATCGTTGTCATCC	PAGE
		R	GCAAATTGTCCTGCTAAGCT	
	c.1975G>C	F	GGCATCATAAGTGATGCTGTTT	PAGE
		R	CCACATCATTTTACTATTGCCAAA	
*MT-RNR1*	m.1555A>G	F	CACGTAAAGACGTTAGGTCAA	PAGE
		R	GAAATCTCCTAAGTGTAAGTTGG	

**Table 3:** The result of OAE hearing screening test in 2174 newborns.

OAE hearing screening	No. of cases	Carrier frequency (%)	*χ* ^2^, *p*
Hearing test (1st)			
Normal	2132	92 (4.32)	0.02, 0.888
Abnormal	42	2 (4.76)	
Hearing test (2nd)			
Normal	20	0 (0)	2.219, 0.231
Abnormal	19	2 (10.5)	

**Table 4:** The display of gene screening and hearing test results in newborns.

Gene name	Mutations	No. of cases	Hearing test (1st)	Hearing test (2nd)
*GJB2*	c.35delG heterozygous	1	Normal	
	c.176_191del16 heterozygous	2	Normal	
	c.235delC heterozygous	46	Normal	
	c.299_300delAT heterozygous	1	Abnormal in both ear	Abnormal in both ear
	c.299_300delAT heterozygous	5	Normal	
*GJB3*	c.538C>T heterozygous	4	Normal	
*SLC26A4*	c.IVS7-2A>G heterozygous	19	Normal	
	c.2168A>G heterozygous	1	Abnormal in both ear	Abnormal in right ear
	c.2168A>G heterozygous	4	Normal	
	c.1174A>T heterozygous	5	Normal	
	c.1226G>A heterozygous	1	Normal	
	c.1975G>C heterozygous	1	Normal	
*MT-RNR1*	m.1555A>G homoplasmy	4	Normal	
	WT	4	Abnormal in both ear	Passed
	WT	7	Abnormal in both ear	Same as 1st
	WT	9	Abnormal in left ear	Passed
	WT	7	Abnormal in left ear	Same as 1st
	WT	7	Abnormal in right ear	Passed
	WT	1	Abnormal in right ear	Same as 1st
	WT	1	Abnormal in both ear	Abnormal in left ear
	WT	1	Abnormal in both ear	Abnormal in right ear
	WT	2	Abnormal in right ear	Lost follow-up
	WT	1	Abnormal in left ear	Lost follow-up

The article "Concurrent Hearing and Genetic Screening among Newborns in Ningbo, China" was retracted in 2023. Reasons: signs of a paper mill; compromised peer review; unreliable results or conclusions.

## Data Availability

The data used to support the findings of this study are available from the corresponding author upon request.

## References

[1] Olusanya B. O., Neumann K. J., Saunders J. E. (2014). The global burden of disabling hearing impairment: a call to action. *Bulletin of the World Health Organization*.

[2] Olusanya B. O. (2012). Neonatal hearing screening and intervention in resource-limited settings: an overview. *Archives of Disease in Childhood*.

[3] Wang Q., Xiang J., Sun J. (2019). Nationwide population genetic screening improves outcomes of newborn screening for hearing loss in China. *Genetics in Medicine*.

[4] Dai P., Huang L. H., Wang G. J. (2019). Concurrent hearing and genetic screening of 180,469 neonates with follow-up in Beijing, China. *American Journal of Human Genetics*.

[5] Hao Z., Fu D., Ming Y. (2018). Large scale newborn deafness genetic screening of 142, 417 neonates in Wuhan, China. *PLoS One*.

[6] Cao S., Sha Y., Ke P., Li T., Yuan W., Huang X. (2020). Deafness gene mutations in newborns in the Foshan area of South China with bloodspot-based genetic screening tests. *American Journal of Audiology*.

[7] He X., Li X., Guo Y. (2018). Newborn screening of genetic mutations in common deafness genes with bloodspot-based gene chip array. *American Journal of Audiology*.

[8] Xiong Y., Zhong M., Chen J., Yan Y. L., Lin X. F., Li X. (2017). Effect of GJB2 235delC and 30-35delG genetic polymorphisms on risk of congenital deafness in a Chinese population. *Genetics and Molecular Research*.

[9] Peng Q., Huang S., Liang Y. (2016). Concurrent genetic and standard screening for hearing impairment in 9317 southern Chinese newborns. *Genetic Testing and Molecular Biomarkers*.

[10] Zhao P., Lin L., Lan L. (2018). Analysis of mutation spectrum of common deafness-causing genes in Hakka newborns in southern China by semiconductor sequencing. *Medicine (Baltimore)*.

[11] Koohiyan M. (2019). A systematic review of SLC26A4 mutations causing hearing loss in the Iranian population. *International Journal of Pediatric Otorhinolaryngology*.

[12] Böttger E. C. (2010). Mutant A1555G mitochondrial 12S rRNA and aminoglycoside susceptibility. *Antimicrobial Agents and Chemotherapy*.

The article "Concurrent Hearing and Genetic Screening among Newborns in Ningbo, China" was retracted in 2023. Reasons: signs of a paper mill; compromised peer review; unreliable results or conclusions.

[13] Lang-Roth R. (2014). Hearing impairment and language delay in infants: diagnostics and genetics. *GMS Current Topics in Otorhinolaryngology - Head and Neck Surgery*.

[14] Li S. X., Chen D. L., Zhao S. B. (2015). Cordblood-based high-throughput screening for deafness gene of 646 newborns in Jinan area of China. *Clinical and Experimental Otorhinolaryngology*.

[15] Wu H., Feng Y., Jiang L. (2016). Application of a new genetic deafness microarray for detecting mutations in the deaf in China. *PLoS One*.

[16] Lu C. Y., Tsao P. N., Ke Y. Y. (2018). Concurrent hearing, genetic, and cytomegalovirus screening in newborns, Taiwan. *The Journal of Pediatrics*.

